The article "Intracoronary Adenosine versus Intravenous Adenosine during Primary PCI for ST-Elevation Myocardial Infarction: Which One Offers Better Outcomes in terms of Microvascular Obstruction?" was retracted in 2013. Reasons: fabricated or falsified data; an official misconduct investigation; misconduct by an author; errors in the data.

# Intracoronary Adenosine versus Intravenous Adenosine during Primary PCI for ST-Elevation Myocardial Infarction: Which One Offers Better Outcomes in terms of Microvascular Obstruction?

**DOI:** 10.1155/2013/248476

**Published:** 2013-03-27

**Authors:** Gemina Doolub, Erica Dall'Armellina

**Affiliations:** ^1^Cardiology Department, John Radcliffe Hospital, Oxford OX3 9DU, UK; ^2^Oxford Centre for Clinical Magnetic Resonance, John Radcliffe Hospital, Oxford, UK

## Abstract

*Aims*. Previous studies have suggested that intravenous administration of adenosine improves myocardial reperfusion and reduces infarct size in ST-elevation myocardial infarction (STEMI) patients. Intracoronary administration of adenosine has shown conflicting results. *Methods*. In this retrospective, single-centre, blinded clinical study, we assessed whether selective intracoronary administration of adenosine distal to the occlusion site immediately before initial balloon inflation reduces microvascular obstruction (MVO) as assessed with cardiac magnetic resonance imaging (MRI). Using contrast-enhanced sequences, microvascular obstruction (MVO) was calculated. We found 81 patients presenting with STEMI within 12 h from symptom onset who were eligible for the study. In 80/81 (100%) patients receiving the study drug, MRI was performed on Day 1 after primary angioplasty. *Results*. The prevalence of MVO was reduced in the patients treated with intracoronary adenosine, (45%) compared to 85% of patients who were administered intravenous adenosine (*P* = 0.0043). We found that the size of MVO in patients receiving intracoronary adenosine was significantly reduced compared to 0.91 g in the intravenous-treated group (*P* = 0.027). There was no statistically significant difference in TIMI flow and clinical outcomes after primary PCI. *Conclusion*. We found significant evidence that selective high-dose intracoronary administration of adenosine distal to the occlusion site of the culprit lesion in STEMI patients results in a decrease in microvascular obstruction.

## 1. Introduction

The concept of “no reflow” refers to a state of myocardial tissue hypoperfusion in the presence of a nonoccluded epicardial coronary artery. The underlying cause of no reflow is microvascular obstruction, which may be produced by various mechanisms [1, 2].

“Reperfusion no reflow” [2] occurs after primary percutaneous coronary intervention (PCI) for reperfusion of an infarct artery in the setting of acute myocardial infarction (AMI) and may be asymptomatic or may present clinically with continued chest pain and ST-segment elevation [3].

Reperfusion no reflow is an independent predictor of adverse clinical outcome after AMI, regardless of infarct size. Despite successful recanalization, perfusion of the ischaemic myocardium is either unrestored or incompletely restored in up to 30% of patients as a result of microvascular obstruction (MVO) [4], which is associated with higher incidence of left ventricular (LV) dysfunction, complications, and death.

Multiple therapies [5] for no reflow have been tested in animals and to a lesser degree in humans. 

Beneficial effects of intracoronary diltiazem, verapamil, epinephrine, nitroprusside, and adenosine have been reported [5–8].

While large randomized trials [4, 5, 9] have suggested that intravenous administration of adenosine during intervention for STEMI may reduce infarct size, especially at higher doses, the effect of intracoronary adenosine in reducing microvascular obstruction is still relatively controversial [9, 10].

 In a trial of 54 patients who underwent primary percutaneous transluminal coronary angioplasty, intracoronary adenosine significantly decreased the rate of noreflow [9]; however, in a later trial of 112 patients undergoing primary PCI with stenting [10, 11], adenosine use was not associated with an improvement in the degree of microvascular obstruction or in a decrease in infarct size at four months [12, 13].

## 2. Study Aims

The aim of this study was to investigate the effect of selective intracoronary administration of adenosine immediately before initial balloon inflation on microvascular obstruction in an unselected population of patients with STEMI.

## 3. Materials and Methods

This study was a single-centre, retrospective, randomized, blinded clinical study with blinded evaluation of endpoints. All consecutive patients presenting with a suspected acute STEMI to a large tertiary referral centre for interventional cardiology in the UK were eligible for the study. Data was collected using our trust local interventional cardiology database (Datacam), electronic discharge summaries, and medical notes. The study was designed and carried out in the Oxford Centre for Clinical Magnetic Resonance Research Centre (OCMR), located at the John Radcliffe Hospital, Oxford. 

Inclusion criteria were as follows:

- symptoms of chest pain suggestive of myocardial ischaemia for at least 20 min,
- a time from onset of symptoms of <12 h,
- an ECG showing ST-segment elevation of >0.1 mV in two or more limb leads or >0.2 mV in two or more contiguous praecordial leads,
- presumed new left bundle-branch block,
- raised troponin (cut-off taken to be troponin >0.04 in Oxford Radcliffe Hospitals NHS Trust),
- patients undergoing primary angioplasty with lesions amenable to stenting,
- patients consenting to MRI within 24 hours of primary angioplasty,
- patients aged >18.

Exclusion criteria were as follows:

- patients receiving intravenous adenosine during the procedure,
- contraindication to heparin, low-molecular-weight heparin, or clopidogrel,
- anticipated difficult vascular access,
- cardiogenic shock,
- inability to give informed consent,
- High-grade atrioventricular block
- severe asthma,
- treatment with theophylline, glibenclamide, or dipyridamole,
- prior coronary artery surgery,
- participation in any investigational drug or device study within the past 30 days,
- contraindications to MRI, for example, an incompatible pacemaker in situ,
- Patients with non-STEMI,
- Patients with ST-elevation MI but absent coronary artery disease angiographically.

## 4. Treatment

After coronary angiography, eligible patients received a bolus injection of intracoronary adenosine (900 micrograms in 5 mL of 0.9% sodium chloride solution). Control patients received an intravenous bolus injection of adenosine (900 micrograms in 20 mL sodium chloride) during the procedure.

After crossing the obstruction of the infarct-related coronary artery with a long guide wire, an over-the-wire balloon (Maverick) was positioned at the level of the obstruction. The guide wire was removed and a small quantity of diluted contrast medium was carefully injected through the central lumen of the balloon catheter to confirm positioning of the catheter tip downstream of the obstruction and to assess patency of the distal vessel. Consequently, the study drug solution was injected by hand through the central lumen of the balloon catheter into the distal vascular bed over 60 seconds. The guide wire was then reinserted through the balloon catheter and advanced to a distal position, and the balloon was inflated. After deflation of the balloon, the procedure was continued per operator preference. As the study was carried out after 2006, we had to ensure that we excluded cases of thrombus aspiration or the use of any other additional device except coronary balloons and stents as per protocol.

All patients received aspirin (300 mg), low-molecular-weight heparin (in the form of dalteparin ACS treatment dose as per patient's weight), and clopidogrel (600 mg) after confirmation of ST-segment elevation on the first ECG. Before commencing primary PCI, patients received a bolus of the glycoprotein IIb/IIIa inhibitor abciximab (0.25 mg/kg), followed by a 12 h infusion. The standard treatment in all patients after primary PCI included aspirin, clopidogrel, *β*-blockers, lipid-lowering agents, and angiotensin-converting enzyme inhibitors.

## 5. Endpoints

The primary endpoint was microvascular obstruction (MVO), which was defined as the very dark region within a bright area of myocardial infarction scar tissue (Figure 2). MVO on MRI at Day 1 was expressed as a percentage of the infarcted area.

Secondary endpoints were TIMI flow grade, major adverse cardiac events at 30 days, left ventricular (LV) function as assessed using MRI at Day 1, and evolution of cardiac markers in the first 24 hours (Figures 3 and 4).

## 6. Cardiac Magnetic Resonance Imaging

Cardiac MRI studies were performed on Day 1 of acute STEMI. Both qualitative and semiquantitative methods were used to assess the extent of early MVO on MRI (Table 2).

On each MRI slice, a region of interest (ROI) was drawn in the centre of the left ventricular (LV) cavity, avoiding papillary muscles.

The three contours (epicardium, endocardium, and blood pool) were copied (registered) to the other images, adjusting for breathing motion.

The myocardium was divided into the relevant segments, using a reference point at the inferior/anterior LV-RV junction. The remaining segments were automatically assigned. The start of the upslope of the time-intensity segment was identified for each slice. The time-intensity curve for each myocardial segment was viewed (Figures 5 and 6).

## 7. Angiographic Analysis

Coronary angiograms obtained before and after primary PCI were reviewed by two experienced interventional cardiologists and a report created on the Datacam software. On the initial angiogram and on the angiogram after stenting, TIMI flow grade was assessed. Site of infarct, door-to-balloon times, medications used during the procedure, and intraprocedural adverse events were also recorded.

## 8. Biomarkers Reflecting Infarct Size

Serum troponin I measurements were collected in all patients during hospitalization. Blood was collected on admission and at 12 hours after revascularization.

## 9. Followup

Followup data at 30 days after primary PCI was collected from hospital records and discharge summaries.

## 10. Acute Adverse Events

These were recorded onto Datacam by the interventional cardiologist performing the procedure.

## 11. Statistical Analysis

Continuous normally distributed variables are presented as mean values and standard deviations. For skewed distributed variables, median values with interquartile range (IQR) are shown. Comparisons between the groups were done by means of an analysis of variance (ANOVA) using randomized treatment and stratum as factors in the model. Subgroup analyses were performed for MVO by age, gender, time to PCI, diabetes, baseline TIMI, final TIMI, and infarct location. All tests were two-sided and assessed at the 5% significance level. In view of the exploratory nature of this study, no correction was applied for multiple testing. Statistical analysis was performed using the SPSS and Excel software, version 2010 for Mac. 

## 12. Results

This study comprised 81 patients who underwent primary PCI for STEMI at the John Radcliffe Hospital, Oxford Radcliffe Hospitals NHS Trust. One patient was excluded from the study, as he could not tolerate MRI scanning due to severe claustrophobia. Of the remaining 80 patients, half (*n* = 40) were given intracoronary adenosine during primary PCI, whereas the remainder (*n* = 40) received intravenous adenosine. Patients randomised to intracoronary adenosine had a higher heart rate on admission compared to patients who had intracoronary adenosine. Patients who received intracoronary adenosine more often had a medical history of diabetes and previous PCI, whereas patients who received intravenous adenosine more often had a history of hypertension and hypercholesterolaemia. TIMI flow 0 or 1 was present in 36 of the 40 patients (90%) having intracoronary adenosine and in 32 of the 40 patients (80%) receiving intravenous adenosine.

All other procedural characteristics did not significantly differ between the two treatment groups—including the stent type and size used, as well as the use of Abciximab (Reopro) infusion during the procedure (Table 1). All patients included in this study had drug-eluting stents (DESs) used during primary PCI.

## 13. Magnetic Resonance Imaging Results

Of the 80 patients included in the study, all underwent MRI during the first 24 hours of admission for primary PCI. Infarct volume was 19.6 g (17.9, 29.9) in the intracoronary-treated patients versus 19.9 g (17.8, 32.4) in the intravenous group of patients (*P* = 0.35) or—expressed as a percentage of the left ventricular mass—19.2% (8.6, 29.7) versus 16.8% (10.9, 22.7) (*P* = 0.11).

Microvascular obstruction (MVO) was observed in 18 of the 40 intracoronary-treated patients (45%) when compared with 34 of the 40 (85%) intravenous treated patients (*P* = 0.0043). The extent of early MVO was 0.35 g (0, 0.53) in the patients receiving intracoronary adenosine and 0.91 g (0.19–1.25) in the intravenous treated group (*P* = 0.027). Expressed as a percentage of the infarct area, this resulted in an MVO of 2.04% (0, 3.75) in the intracoronary group, compared to 7.83% (2.85, 12.13) in the intravenous group (*P* = 0.0014) (Figure 1).

This treatment effect was present in both strata, irrespective of time of symptom onset. Other MRI analyses were comparable between the two treatment groups, with the exception of a higher ejection fraction in the coronary-treated patients.

Additional analyses, adjusted for baseline TIMI, diabetes, time to PCI, and infarct location, were performed for the main endpoints of interest. Subgroup analyses for microvascular obstruction (MVO) revealed a statistically significant interaction between treatment and baseline TIMI flow grade (0/1 versus 2/3) (*P* = 0.042), whereby a statistically significant treatment benefit of intracoronary adenosine was found for patients with TIMI 2/3 at baseline (*P* = 0.037). A similar beneficial effect of treatment was found in the group of patients with TIMI flow grade 0/1 at baseline, but this difference was not statistically significant (*P* = 0.068).

## 14. Angiographic Results

After primary PCI, TIMI flow grade 3 was present in 40 of the 40 patients (100%) receiving intracoronary adenosine and in 36 of the 40 patients (90.0%) receiving intravenous adenosine (*P* = 0.077; Table 3). 

## 15. Biomarkers

Calculation of the area under the curve of cardiac markers as an estimation of infarct size was not performed if either the first or last measurement was missing. Other missing values were imputed by linear interpolation. The area under the curve for troponin I could only be calculated for 78 of the 80 patients and showed no significant differences between treatment groups (Table 4), irrespective of time from symptom onset. One major limitation in the measurement of troponin was the fact that the assay used by the Oxford Hospitals Trust did not enable measurements of troponin, which meant that any troponin value exceeding this range was consistently reported as being >50.

## 16. Complications during Primary PCI

An increase of chest pain during or immediately after selective administration of adenosine 900 micrograms distally to the occlusion site was not observed at all. Occlusion of a significant side branch, no reflow phenomenon, bradycardia, ventricular tachycardia, and ventricular fibrillation were not seen in either of the two treatment groups. Dissection was numerically more frequent in the intravenous group of patients compared with patients receiving intracoronary adenosine, the difference, however, not reaching statistical significance (2/40 (5%) versus 0/40 (1.9%), *P* = 0.87). The incidence of second- and third-degree atrioventricular block was also numerically higher in the intravenous group of patients (4/40 (10%) and 2/40 (5%)) than in intracoronary-treated patients (2/40 (5%) 0/40 (0%)). These conduction blocks disappeared within 4 minutes, without clinical sequelae (Table 5).

## 17. Clinical Outcomes

None of the patients died during initial hospitalization: one patient from the control group developed heart block 9 hours after stenting of the right coronary artery (RCA), which required urgent pacing.

Between discharge and 30-day followup, an additional patient randomized to intravenous adenosine developed a recurrent myocardial infarction at 28 days, for which he underwent repeat coronary angioplasty.

At 30 days, none of the patients had died in each treatment group.

## 18. Discussion

This retrospective, blinded, case-controlled clinical study demonstrated that selective intracoronary administration of adenosine distally to the occlusion site and immediately before initial balloon inflation improved reperfusion in patients with STEMI. There were significant differences in MVO and TIMI flow as assessed by angiography and MRI. However, there were no significant difference in enzymatic infarct size and clinical outcome at 30 days after primary PCI between patients given intracoronary adenosine, as compared to the control group. 

In the present study, we attempted to avoid some of the methodological limitations of earlier trials [11–13]. First, we used MRI to assess the primary endpoint, microvascular obstruction, because it is less influenced by differences in the extent of ischaemic myocardium at baseline. Second, all study personnel remained blinded to treatment assignment until completion of all analyses. Third, the study drug was consistently administered subselectively to the ischaemic myocardium, prohibiting inadvertent spillover into other coronary branches. Fourth, we used a consistently high dose of adenosine, 900 micrograms, proven to be safe and well tolerated. We also directly compared the effects of intracoronary versus intravenous adenosine, which has not been done in previous studies. Finally, in each case the intracoronary adenosine was consistently administered before initial balloon inflation.

One may argue that the presence of a beneficial effect of intracoronary adenosine is due to differences in baseline clinical characteristics, favouring intracoronary-treated patients. However, there were no significant differences in baseline characteristics between the two treatment groups with the exception of a slightly higher heart rate on admission in patients who received intracoronary adenosine and a higher incidence of diabetes mellitus and previous PCI in the same group of patients. On the contrary, such differences should logically have favoured the intravenous group, thus inducing smaller amounts of MVO—which was clearly not the case in this study.

## 19. Limitations of the Study

First, the primary endpoint was MVO and we cannot comment on clinical endpoints, for which the study was underpowered. Second, 28% of patients had limited spontaneous reperfusion before intracoronary administration of the study drug and in a few more mere passage of the guide wire may have mediated some degree of reperfusion. Hence, in these patients, adenosine was not truly given before reperfusion. However, for MVO, we identified a large interaction between treatment and baseline TIMI, whereby a statistically significant treatment benefit of intracoronary adenosine was found for patients with TIMI 2/3 flow at baseline and a nonstatistically significant benefit was found for the TIMI 0/1 group. At this stage, it is not very clear to us how this finding can be explained. Third, the trial included a significant proportion of patients with small and/or completed infarcts. Fourth, infarct size cannot be reliably assessed when biomarkers are drawn every 8 h as in this study. And finally, intracoronary adenosine boluses may be too short acting for any beneficial effect and we cannot exclude the efficacy of prolonged intracoronary administration.

## 20. Conclusions and Implications

We found convincing evidence that selective intracoronary administration of high-dose adenosine as adjunctive therapy to primary PCI reduces MVO in patients with STEMI. Future attempts at improving myocardial reperfusion, preventing reperfusion injury, and salvaging ischaemic myocardium should focus on finding the optimal dose of intracoronary adenosine that should be used in order to create a maximum beneficial effect.

## Figures and Tables

**Figure 1:** Microvascular obstruction: three-chamber MRI demonstrates near full-thickness transmural infarct (arrow) in the basal anteroseptum. There is a black area (curved arrow) within the bright scar consistent with microvascular obstruction [14].

**Figure 2:** Delineation and calculation of MVO by drawing the relevant contours: white area demonstrates the area of infarct, while the black area within shows the extent of microvascular obstruction (MVO).

**Figure 3:** Left ventricle before contrast.

**Figure 4:** Left ventricle after contrast.

**Figure 5:** Myocardial time-intensity curve.

**Figure 6:** Box plot showing microvascular obstruction (%) (primary endpoint). Box plot shows median and interquartile range. *Q*1, *Q*3 = first and third quartile, *IQR* = *Q*3 − *Q*1. “+” sign indicates mean value.

**Table 1:** Baseline patient characteristics (% in brackets).

Characteristic	Intracoronary adenosine (*n* = 40)	Intravenous adenosine (*n* = 40)
Age (years)	61.0	59.8
Male gender	30 (75)	32 (80)
Heart rate (b.p.m.)	96	87
Systolic blood pressure (mm Hg)	156	162
Diastolic blood pressure (mm Hg)	98	104
Current smoker	26 (65)	30 (75)
History		
Myocardial infarction	6 (15)	4 (10)
Diabetes mellitus	6 (15)	2 (5)
PCI	4 (10)	2 (5)
Family history	12 (30)	10 (25)
Hypertension	18 (45)	22 (55)
Hypercholesterolaemia	12 (30)	22 (55)
Door-to-balloon time (median, IQR), min	16.1	15.8
Angiographic		
Infarct-related vessel		
RCA	20 (50)	22 (55)
LAD	18 (45)	16 (40)
Cx	2 (5)	2 (5)
TIMI flow before PCI		
0	32 (80)	20 (50)
1	4 (10)	12 (30)
2	4 (10)	8 (20)
3	0 (0)	0 (0)
0/1	36 (90)	32 (80)
2/3	4 (10)	8 (20)
Stent diameter, mm	3.0	3.0
Stent length, mm	19.5	21.7
GPIIb/IIIa inhibitor during PCI	40 (100)	40 (100)

**Table 2:** Magnetic resonance imaging results at Day 1.

	Intracoronary adenosine (*n* = 40)	Intravenous adenosine (*n* = 40)	*P* value
Myocardial evaluation (median, IQR)			
Microvascular obstruction present	18/40 (45%)	34/40 (85%)	0.0043
Microvascular obstruction (g)	0.35 (0, 0.53)	0.91 (0.19, 1.25)	0.027
Microvascular obstruction (%)	2.04 (0, 3.75)	7.83 (2.85, 12.13)	0.0014
Infarct volume (g)	19.60 (17.9, 29.9)	19.90 (17.8, 32.4)	0.35
Infarct volume (% LV mass)	19.20 (8.6, 29.7)	16.80 (10.9, 22.7)	0.11
LV function (mean, SD)			
SV (mL)	23.81 (11.10)	24.42 (14.31)	0.44
EF (%)	31.54 (11.49)	29.40 (10.15)	0.27
LV mass (g)	70.40 (24.8)	99.89 (22.3)	0.35

**Table 3:** TIMI flow grade following primary PCI.

	Adenosine	Control	*P* value
TIMI flow grade			
0	0	0	
1	0	4	
2	0	0	
3	40	36	0.077
0/1	0	4	0.068
2/3	40	36	0.037

**Table 4:** Infarct based on cardiac markers (median (interquartile range)).

	Intracoronary adenosine	Intravenous adenosine	*P* value
Troponin I maximum (microg/L)	50 (32.4; 50) (*n* = 19)	50 (23.5; 50) (*n* = 20)	0.31
Troponin AUC (microg/L × h)	400 (296.8; 400) (*n* = 19)	400 (196.1; 400) (*n* = 20)	0.28

**Table 5:** Complications during primary percutaneous coronary intervention [*n* (%)].

Complication during/immediately after PCI	Intracoronary adenosine (*n* = 40)	Intravenous adenosine (*n* = 40)	*P* value
Increase of chest pain during study drug administration	0 (0%)	0 (0%)	0.91
Occlusion of side branch ≥ 2 mm	0 (0%)	0 (0%)	0.76
Distal embolization	0 (0%)	0 (0%)	0.76
No reflow	0 (0%)	0 (0%)	1.53
Dissection	0 (0%)	2 (5%)	0.27
Second-degree AV block	2 (5%)	4 (10%)	0.63
Third-degree AV block	0 (0%)	2 (5%)	0.75
VT (ventricular tachycardia)	0 (0%)	0 (0%)	0.57
VF (ventricular fibrillation)	0 (0%)	0 (0%)	0.98

## Abbreviations

ACS: Acute coronary syndrome
Cx: Circumflex artery
LAD: Left anterior descending artery
MRI: Magnetic imaging resonance
MVO: Microvascular obstruction
PCI: Percutaneous coronary intervention
RCA: Right coronary artery
STEMI: ST-elevation myocardial infarction
TIMI: Thrombolysis in myocardial infarction.
